The article "Examination of the effects of microRNA-145-5p and phosphoserine aminotransferase 1 in colon cancer" was retracted in 2026. Reasons: concerns about the data; concerns about the results or conclusions.

# Examination of the effects of microRNA-145-5p and phosphoserine aminotransferase 1 in colon cancer

**DOI:** 10.1080/21655979.2022.2071010

**Published:** 2022-05-26

**Authors:** Ruliang Ding, Weiwen Hong, Liang Huang, Jinfan Shao, Wenfeng Yu, Xijuan Xu

**Affiliations:** Department of Anorectal Surgery, Taizhou First People’s Hospital, Taizhou, Zhejiang Province, China

**Keywords:** Colon cancer, microRNA-145-5p, PSAT1, proliferation, cell cycle

## Abstract

Previous studies manifested that microRNA-145-5p is pivotal in the development of various cancers. Nevertheless, the potential function of microRNA-145-5p in colorectal cancer remains unclear. This study attempted to investigate the potential role and possible mechanism of microRNA-145-5p in colon cancer. MicroRNA-145-5p and phosphoserine aminotransferase 1 (PSAT1) levels in colon cancer cells were assayed via quantitative reverse transcription polymerase chain reaction (qRT-PCR). Cell proliferation and cell cycle status were assessed using Cell Counting Kit-8, colony formation, and flow cytometry. The target binding relationship of microRNA-145-5p and PSAT1 was identified using bioinformatics analysis and dual-luciferase reporter gene assay. The result of qRT-PCR disclosed that microRNA-145-5p was markedly down-regulated and PSAT1 level was up-regulated in colon cancer cell lines. Besides, enforced microRNA-145-5p level repressed proliferation of colon cancer cells, and cells were arrested in G0-G1 phase. Bioinformatics analysis and dual-luciferase reporter genes confirmed that PSAT1 was a downstream target of microRNA-145-5p. Enforced PSAT1 level remarkably modulated cell cycle and fostered cell proliferation. Furthermore, rescue experiments displayed that microRNA-145-5p restrained cell cycle progression and cell proliferation and forced PSAT1 level could partially reverse this process. Taken together, our findings demonstrated that microRNA-145-5p repressed colon cancer cell cycle progression and cell proliferation via targeting PSAT1. Our findings identified microRNA-145-5p as an essential tumor repressor gene in colon cancer and may provide a novel biomarker for colon cancer.

## 1. Introduction

Colon cancer has attracted the attention of humans due to its high morbidity and mortality worldwide [1,2]. As the rise of people’s living standard, the change of diet structure, the morbidity of colon cancer shows a rising trend year by year. Given that the exact pathogenesis of colon cancer has not yet been fully clarified [3,4], surgical treatment, neoadjuvant chemoradiotherapy, postoperative chemotherapy and other traditional treatment methods are still common treatment approaches [5]. To develop effective therapeutic strategies for colon cancer, what the most important is to further understand the molecular mechanism that causes colon cancer.

MicroRNAs are endogenous non-coding RNAs with an average length of mature microRNAs being 22 nucleotides. By complementary pairing with the 3’-untranslated region (3’-UTR) within target mRNA, miRNAs destabilize mRNA or prevent translation to achieve gene silence [6,7]. It is reported that miRNAs are pivotal in regulation of cancer progression in colon cancer [8]. For example, microRNA-6716-5p targets N-acetyltransferase 10 to facilitate cell migration and invasion in colon cancer [9]. MicroRNA-664b-3p regulates colon cancer tumor growth progression by repressing benzimidazole 3 protein level [10]. MicroRNA-301b-3p accelerates colorectal cancer cell proliferation and migration by targeting homeobox B1 [11]. MicroRNA-145-5p was proven to be a repressor in varying cancer cells [12–14], but the modulatory mechanism of microRNA-145-5p in colon cancer cells has not been reported.

Phosphoserine aminotransferase 1 (PSAT1) participates in cell proliferation *in vitro* [15–17]. Serine takes a crucial part in the synthesis of biomolecules that hasten cell proliferation [18–20]. Recent evidence suggested that serine overactivation contributes to tumorigenesis [21]. PSAT1 was found to be upregulated in ovarian cancer, breast cancer, and non-small cell lung cancer, enhancing cell proliferation, metastasis and chemical resistance, all of which result in poor prognosis [15,16,22]. Other studies found that PSAT1 mRNA is upregulated with colon cancer progression [23,24]. But, the correlation between PSAT1 and microRNA-145-5p in colon cancer is warranted.

In this work, we hypothesized that microRNA-145-5p may play an essential role in colon cancer progression. This study aimed to investigate the effect of the microRNA-145-5p/PSAT1 axis on the proliferation and cycle of colon cancer cells. Therefore, based on bioinformatics analysis and a series of biological experiments, we found that microRNA-145-5p was underexpressed in colon cancer, and the expression of PSAT1, which is a downstream target of microRNA-145-5p, was up-regulated. MicroRNA-145-5p targeted PSAT1 to hinder cycle progression in colon cancer. Our study provides a new avenue for colon cancer treatment.

## 2. Materials and methods

### 2.1. Bioinformatics analysis

Colon cancer-related expression data of miRNA (normal sample: 8, tumor sample: 450) and mRNA (normal sample: 41, tumor sample: 473) was accessed from The Cancer Genome Atlas (TCGA) database. The gene expression differences between normal group and the tumor group of miRNA and mRNA were analyzed by using the ‘edgeR’ package (|logFC|>2, adj.pvalue<0.05). Downstream target genes for the miRNA of interest were identified by miRDB, starBase and miRTarBase databases, and potential mRNAs with binding sites of microRNA-145-5p were determined. Correlation analysis was conducted for candidate mRNAs with microRNA-145-5p to identify the mRNA the most likely to be downstream target gene of microRNA-145-5p.

### 2.2. Cell culture

In this study, a total of 6 cancer cell lines were used for experiments. Human colon cancer cell lines Caco-2 (BNCC102170), LoVo (BNCC338601), HT29 (BNCC100164), SW480 (BNCC100604), SW620 (BNCC100162) and human normal epithelial cell line NCM460 (BNCC339288) were accessed from BeNa Culture Collection. All cells were incubated in Dulbecco’s modified Eagle’s medium (sigma, USA) with 10% fetal bovine serum (GE Healthcare Life Sciences, USA) at 37°C with 5% CO_2_ [25].

### 2.3. Quantitative reverse transcription polymerase chain reaction (qRT-PCR)

Total RNA in colon cancer cells was isolated using Trizol (Invitrogen, USA). Complementary DNA (cDNA) for mRNA and miRNA were synthesized using the PrimeScript™ RT Reagent Kit (Takara, Japan) and Transscript® miRNA First-Strand cDNA Synthesis SuperMix Kit (Full Golden Bio, China), respectively. Then, qRT-PCR was run with TB Premix Ex Taq (Takara, Japan). The primer sequences listed in Table 1 were synthesized by Sangon Biotech (China). MicroRNA-145-5p and PSAT1 levels were referred to U6 and *β*-actin, respectively. 2^−ΔΔCt^ method [26] was employed to obtain relative RNA expression. The assay was repeated 3 times.

**Table 1.** qRT-PCR primer sequences

Target gene	Primer (5’-3’)
microRNA-145-5p	F: 5’-GTCCAGTTTTCCCAGGAATC-3’
	R: 5’-AGAACAGTATTTCCAGGAAT-3’
U6	F: 5’-CTCGCTTCGGCAGCACA-3’
	R: 5’-AACGCTTCACGAATTTGCGT-3’
PSAT1	F: 5’-TGCCCAGAAGAATGTTGGCT-3’
	R: 5’-TCCAGAACCAAGCCCATGAC-3’
*β*-actin	F: 5’-GATTCCTATGTGGGCGACGAG-3’
	R: 5’-CCATCTCTTGCTCGAAGTCC-3’

### 2.4. Cell transfection

Mimic NC, microRNA-145-5p mimic, inhibitor NC and microRNA-145-5p inhibitor were purchased from Sangon (China). Lipofectamine 2000 (Thermo Fisher Scientific,USA) was introduced to transiently transfect them into cell line HT29. oe-NC and oe-PSAT1 were constructed using lentiviral vector pLVX-IRES-neo (Clontech, USA). To knock out PSAT1, PSAT1-targeted sh-RNA (GeneChem Co. Ltd., China) was spliced into GV248 lentivirus plasmids which were then transfected into cell line HT29. The sh-RNA primer sequence is as follows: 5’ -ACTCAGTGTTGTTAGAGAT-3’. All cells were grown in complete medium for 24 h before transfection. Before transient transfection, the cells should be washed with PBS (pH 7.4) [11].

### 2.5. Cell Counting Kit-8 (CCK-8)

Changes in cell proliferation were assessed using the CCK-8 assay as previously described [27]. The cell concentration was controlled at 2 × 10^3^ cells/mL, and then the cells were inoculated in a 96-well plate for proliferation examination after resuspension. At 24, 48, 72, and 96 h, cells were cultured with 10 μL CCK-8 reagent (Shanghai Biotech Institute, China) for another 2 h. Finally, the absorbance at 450 nm was evaluated using a microtiter plate reader (Thermo Fisher Scientific, USA). The assay was repeated 3 times independently.

### 2.6. Colony formation assay

Changes in cell proliferation were assessed using colony formation assays as previously described [28]. Colon cancer cells (1 × 10^3^) were resuspended and then seeded into a 6-well plate. The cells were incubated at 37°C for 2 weeks to assess cell proliferative potential. Next, cells were fixed with 4% paraformaldehyde for 20 min, immediately stained with 0.1% crystal violet for 20 min, and then photographed for observation of cell colonies.

### 2.7. Western blot assay

The relevant steps of protein extraction and Western Blot were carried out with reference to the steps of the aforementioned article [25]. Total proteins were extracted from the cells using radioimmunoprecipitation assay lysis buffer (Solarbio, China), and the protein concentrations were measured by bicinchoninic acid protein kit (Beyotime, China). Proteins were isolated and then transferred to a polyvinylidene fluoride membrane by electrophoresis. Then, the membrane was sealed with Tris Buffered Saline Tween with 5% bovine serum albumin. After that, the membrane was then maintained overnight at 4°C with primary rabbit monoclonal antibodies, including PSAT1 (ab96136, 1:500), Cyclin C (ab85927, 1:2000), Cyclin D1 (ab40754, 1:200), Cyclin E1 (ab33911, 1:1000), and β-actin (ab115777, 1:200). Subsequently, the membrane was incubated with Horseradish peroxidase-labeled secondary antibody goat anti-rabbit IgG (ab6721, 1:2000) for 1 h at room temperature. Finally, protein expression visualization was conducted using enhanced chemiluminescence kit (Beyotime, China).

### 2.8. Dual-luciferase reporter assay

The PSAT1 3’-untranslated region (3’-UTR) containing wild-type (WT) or mutant (MUT) binding sites of microRNA-145-5p was ligated into pmiRGLO (Promega, USA) plasmid vectors. Then, plasmids containing WT PSAT1 3’-UTR or MUT PSAT1 3’-UTR were co-transfected into cell line HT29 with mimic NC or microRNA-145-5p mimic to verify the targeting relationship between miRNA and mRNA. After 48 h, luciferase activity was assessed on the luciferase reporter assay system (Promega). Renilla luciferase was employed as internal reference [27]. The assay was repeated 3 times.

### 2.9. Flow cytometry assay

Flow cytometry (BD Biosciences, San Jose, USA) was applied to assess cell cycle [29]. Colon cancer cells were resuspended in 75% ethanol solution, fixed overnight at 4°C, and labeled with prodium iodide/RNase staining buffer for 30 min before detection.

### 2.10. Data analysis

The data were processed and analyzed by GraphPad Prism 8.0 version. All data were presented in mean ± standard deviation. The *t*-test was selected to analyze the differences in data between two groups. When *p* < 0.05, the data difference between groups was viewed statistically significant.

## 3. Results

In this study, we speculated that microRNA-145-5p may play an essential role in colon cancer progression. This study attempted to investigate the effect of microRNA-145-5p/PSAT1 on colon cancer proliferation and cycle. Thus, low expression of microRNA-145-5p in colon cancer was assayed by qRT-PCR, and PSAT1 level was up-regulated. Bioinformatics and dual-luciferase reporter experiments identified PSAT1 as a downstream target of microRNA-145-5p. The effects of microRNA-145-5p and PSAT1 on colon cancer cell cycle and proliferation were detected by CCK-8, colony formation, and flow cytometry. The results manifested that microRNA-145-5p restrained colon cancer cell cycle progression and proliferation, and PSAT1 fostered colon cancer cell cycle progression and cell proliferation. Rescue experiments displayed that microRNA-145-5p repressed cell cycle progression and cell proliferation and enforced PSAT1 expression could partially reverse this process. Taken together, our findings demonstrated that microRNA-145-5p restrained colon cancer cell cycle progression and cell proliferation via targeting PSAT1.

### 3.1. MicroRNA-145-5p is lowly expressed in colon cancer

Isoform Expression Quantification data of colon cancer-related miRNA were obtained from TCGA database, and then 326 differential miRNAs were obtained through differential analysis by ‘edgeR’ (Figure 1(a)). Among them, microRNA-145-5p was conspicuously downregulated in colon cancer tissue (Figure 1(b)). Based on expression data and clinical data of microRNA-145-5p in colon cancer in TCGA database, we manifested that microRNA-145-5p level was noticeably associated with lymph node metastasis, distant metastasis, and disease stage (Supplementary Figure 1). It is confirmed that microRNA-145-5p is downregulated in many cancers [30–32]. The expression status of microRNA-145-5p in cell lines was tested via qRT-PCR, revealing that it was lower in Caco-2, LoVo, HT29, SW480, and SW620 cell lines than that in NCM460 cell line (Figure 1(c)). Then, HT29 cell line with the most obvious expression difference was selected for subsequent cell function experiments.

**Figure 1.** MicroRNA-145-5p is decreased in colon cancer. (a) Volcano map of 326 differential miRNAs (upregulated in red while downregulated in green); (b) Differential expression of microRNA-145-5p in colon cancer and normal tissue samples (blue: normal; Orange: tumor); (c) MicroRNA-145-5p level in human normal colon epithelial cell line and colon cancer cell lines; * denotes *p* < 0.05.

### 3.2. MicroRNA-145-5p suppresses the growth of colon cancer cells and affects cell cycle

Then, the biological functions of microRNA-145-5p in colon cancer cells were explored. Colon cancer cell line HT29 was taken to transfect with microRNA-145-5p mimic, inhibitor and the corresponding controls. The qRT-PCR results uncovered that the microRNA-145-5p expression in microRNA-145-5p mimic group was notably increased compared with mimic NC group, while that in microRNA-145-5p inhibitor group was remarkably decreased compared with inhibitor NC group (Figure 2(a)). Cell colony assay displayed that the rate of colony formation was prominently reduced after upregulating microRNA-145-5p (Figure 2(b)). Meanwhile, the effect of microRNA-145-5p on the activity of colon cancer cells was further verified by CCK-8 assay. Compared with control group, overexpressed microRNA-145-5p markedly inhibited cell proliferative viability, while restrained microRNA-145-5p led to the opposite result (Figure 2(c)). In addition, the flow cytometry results expressed that compared with mimic NC group, the number of cells in G_0_-G_1_ phase of microRNA-145-5p mimic group was notably increased; compared with inhibitor NC group, the proportion of cells in G_0_-G_1_ phase was noticeably decreased in microRNA-145-5p inhibitor group (Figure 2(d)). These results proved that the upregulation of microRNA-145-5p could inhibit proliferation of colon cancer cells and affect the cell cycle progression.

**Figure 2.** MicroRNA-145-5p restrains cell proliferation in colon cancer and affects cell cycle. (a) MicroRNA-145-5p level in HT29 cells with microRNA-145-5p mimic/inhibitor in each treatment group; (b) The colony forming property of HT29 cells in treatment groups; (c) Cell viability of HT29 cells in treatment groups; (d) Cell cycle of HT29 cells in treatment groups; * denotes *p* < 0.05.

### 3.3. MicroRNA-145-5p targets PSAT1

The mRNA expression data in colon cancer were downloaded from TCGA in this study, and then 2,069 differential mRNAs were gained (Figure 3(a)). Next, the miRDB, starBase and miRTarBase databases were introduced to screen target genes of microRNA-145-5p. The predicted results were intersected with the 1,166 differentially upregulated mRNAs to acquire 3 differential mRNAs with targeted binding sites of microRNA-145-5p (Figure 3(b)). Pearson correlation analysis of microRNA-145-5p and these 3 mRNAs denoted that PSAT1 was inversely correlated with microRNA-145-5p and had the highest correlation coefficient (Figure 3(c)). It was also noted that PSAT1 was conspicuously overexpressed in colon cancer tissue (Figure 3(d)). It was confirmed that PSAT1 expression is enforced in tumor tissue and is related to cancer cell proliferation [15,33]. To verify the accuracy of the predicted data, PSAT1 expression was measured in both colon cancer and normal colon epithelial cells. As depicted in Figure 3(e,f), PSAT1 level was prominently increased in colon cancer cells compared to that in normal cells, indicating that PSAT1 was increased in colon cancer.

**Figure 3.** MicroRNA-145-5p targets and binds to PSAT1. (a) Volcano map of differential mRNAs in normal group and tumor group in colon cancer data set (red for upregulated and green for downregulated); (b) Venn plot of predicted target mRNAs of microRNA-145-5p and differentially up-regulated mRNAs; (c) Pearson correlation analysis of microRNA-145-5p and PSAT1; (d) Relative expression of PSAT1 in TCGA (blue: normal and Orange: tumor); (e) PSAT1 mRNA level in different cell lines; (f) PSAT1 protein level in different cells; (g-h) The effect of overexpressed/silenced microRNA-145-5p on PSAT1 level; (i) The binding of microRNA-145-5p to PSAT1; * denotes *p* < 0.05.

Then, changes in PSAT1 expression were detected in cells transfected with mimic NC, microRNA-145-5p mimic, inhibitor NC, and microRNA-145-5p inhibitor (Figure 3(g,h)). Compared with NC group, PSAT1 expression in microRNA-145-5p mimic group was notably decreased, while that in microRNA-145-5p inhibitor group was markedly increased.

Subsequently, the putative-binding sites of microRNA-145-5p on the 3’-UTR of PSAT1 mRNA was confirmed by dual-luciferase reporter gene analysis (Figure 3(i)). Compared with NC group, luciferase activity was inhibited by the co-transfection with microRNA-145-5p mimic and PSAT1-3’-UTR-WT; but there was no notable difference in luciferase activity when cells were co-transfected with microRNA-145-5p mimic and PSAT1-3’-UTR-MUT. The results indicated that there were specific binding sites for microRNA-145-5p on the 3’-UTR of PSAT1, suggesting that PSAT1 was the target gene of microRNA-145-5p in colon cancer.

### 3.4. PSAT1 regulates colon cancer cell cycle and affects cell proliferation

PSAT1 was notably boosted in colon cancer tissue. It is reported that PSAT1 level is enforced in tumor tissue and is related to cancer cell proliferation [15,33]. GSEA pathway enrichment analysis results indicated that PSAT1 was markedly abundant in the cell cycle signaling pathway (Figure 4(a)), while cell cycle signaling pathway is closely related to cancer cell proliferation [34].

**Figure 4.** PSAT1 regulates colon cancer cell cycle and affects cell proliferation. (a) GSEA enrichment analysis for PSAT1. (b-c) PSAT1 mRNA and protein levels in cells with overexpressed/silenced PSAT1. (d-e) The effects of PSAT1 overexpression/silence on cell proliferation. (f) Cell cycle analysis. * denotes *p* < 0.05.

To clarify the function of PSAT1 in colon cancer cells, HT29 cells were infected with specific shRNA to construct cell line silencing PSAT1. Meanwhile, HT29 cells with stably overexpressed PSAT1 were established using PSAT1 overexpression vectors. Then, the mRNA and protein levels of PSAT1 in these cells were examined via qRT-PCR and western blot. The results revealed that PSAT1 was discernibly knocked down in sh-PSAT1 group but increased in oe-PSAT1 group relevant to the control group (Figure 4(b,c)).

After that, CCK-8 assay uncovered that, in comparison to cells in corresponding control groups, the rate of colony formation of HT29 cells was boosted and cell proliferation was accelerated after the expression of PSAT1 was stimulated, while the colony forming ability and proliferative viability of these cells were greatly suppressed after PSAT1 silence (Figure 4(d,e)).

Next, the relationship between PSAT1 and the cell cycle of colon cancer cells was analyzed by flow cytometry. Compared with the control group, overexpressed PSAT1 notably fostered the proportion of cells in S phase and hampered the percentage of cells in G_0_-G_1_ phase. However, inhibition of PSAT1 resulted in a prominent increase in G_0_-G_1_ phase and a notable decrease in the proportion of cells in S phase (Figure 4(f)).

Concludingly, the findings indicated that overexpressed PSAT1 shortened the G_1_ phase of the cell cycle and advanced cells into S phase, thereby enhancing the proliferation of colon cancer cells. Endogenous silencing of PSAT1 blocked colon cancer cells from entering S phase, thereby inhibiting cell proliferation *in vitro*.

### 3.5. MicroRNA-145-5p targets PSAT1 to modulate cell cycle and inhibit cell proliferation of colon cancer

It was previously verified that PSAT1 was upregulated in colon cancer cells and inversely modulated by microRNA-145-5p. In this section, to further identify the binding of microRNA-145-5p and PSAT1, rescue experiments were conducted. Firstly, mimic NC+oe-NC, microRNA-145-5p mimic+oe-NC, and microRNA-145-5p mimic+oe-PSAT1 were transfected into colon cancer cell line HT29, respectively. PSAT1 mRNA and protein levels in each group were assayed through qRT-PCR and western blot (Figure 5(a,b)). According to the results, PSAT1 level in cells was markedly hampered upon overexpressed microRNA-145-5p alone while restored similar to that in the control group after the concurrent upregulation of microRNA-145-5p and PSAT1.

**Figure 5.** MicroRNA-145-5p targets PSAT1 to restrain cell proliferation of colon cancer. a. PSAT1 mRNA level in transfected cells; b. Protein expression of PSAT1, Cyclin c, Cyclin D1 and Cyclin E1 in each group; c-d. The cell proliferation of each transfection group; e. Cell cycle analysis performed on transfected HT29 cells; * denotes *p* < 0.05.

CCK-8 assay result (Figure 5(c)) illustrated that overexpressed microRNA-145-5p markedly inhibited the proliferative viability of cancer cells, while the viability was notably restored in the microRNA-145-5p mimic+oe-PSAT1 group. Meanwhile, the cell colony formation assay (Figure 5(d)) also proved that: enforced expression of microRNA-145-5p restrained cell proliferation, which was remarkably reversed after PSAT1 expression was restored, basically the same as that of the control group. Subsequently, flow cytometry was conducted (Figure 5(e)). The results presented that the proportion of cells in G_0_-G_1_ phase raised prominently in the microRNA-145-5p mimic+oe-NC group while then decreased slightly in the microRNA-145-5p mimic+oe-PSAT1 group. In addition, the expression of cyclin-related proteins (Cyclin C, Cyclin D1, Cyclin E1) in colon cancer cell HT29 in each group was determined by western blot (Figure 5(b)). Compared with microRNA-145-5p mimic+oe-NC group, the levels of cell cycle-related proteins in microRNA-145-5p mimic+oe-PSAT1 group were notably increased. Taken together, microRNA-145-5p regulated cell cycle through PSAT1 to inhibit colon cancer cell proliferation.

## 4. Discussion

In China, the morbidity of colon cancer, one of the gastrointestinal malignancies, is increasing rapidly, and its morbidity as well as mortality closely follows that of lung cancer which has the highest incidence in China. Unfortunately, many unanswered questions remain about the pathogenesis and etiology of colon cancer. In this study, bioinformatics analysis revealed that microRNA-145-5p level in colon cancer tissue was relatively low to that in normal tissue. Differential expression of microRNA-145-5p is thought to be pivotal in cancer cells. According to the current research results, microRNA-145-5p is decreased in a number of cancers, indicating that microRNA-145-5p acts as a tumor repressor gene in cancer cells. For example, microRNA-145-5p restrains prostate cancer cell migration, invasion, and metastasis, and promote cell apoptosis by directly targeting phospholipase D 5 [35]. MicroRNA-145-5p is a tumor repressor in colon cancer, which restrains chemokine (C-X-C motif) ligand 1 and integrin α2 [36]. MicroRNA-145-5p can also inhibit the migration, invasion and epithelial–mesenchymal transition of esophageal squamous cell carcinoma cells through specificity protein 1/nuclear factor κB signaling pathway, so as to be an anti-tumor gene [13].The above research results all confirm that microRNA-145-5p can resist cell growth in cancer. Similarly, here, microRNA-145-5p was found decreased in colon cancer cells, the most obvious in the colon cancer cell line HT29. To clarify the role of microRNA-145-5p in colon cancer pathogenesis, we conducted bioinformatics analysis and cell function experiments. As analyzed, we revealed that microRNA-145-5p may modulate mRNA level of one of its downstream genes, PSAT1. We focused on regulatory relationship between microRNA-145-5p and PSAT1, which may furnish a novel regimen for colon cancer management.

PSAT1 is associated with cell proliferation *in vitro* [24,37]. Earlier studies showed that PSAT1 is vital in cell proliferation. For example, Possemato *et al.* [38] demonstrated that PSAT1 reduction can constrain proliferation of breast cancer cells (BT-20 and MDA-MB-468). Chan *et al.* [39] conducted an immunohistochemistry analysis on 104 cases with non-small cell lung cancer and displayed that PSAT1 level in tumor tissue is higher than that in adjacent normal tissue, and increased PSAT1 is implicated in unfavorable prognosis of patients with early adenocarcinoma. Consistent with previous studies, PSAT1 here was remarkably upregulated in colon cancer cells, and *in vitro* cell experiments indicated that overexpressed PSAT1 fostered colon cancer cell proliferation. We displayed that after microRNA-145-5p was upregulated, the expression of proteins related to cell cycle, such as Cyclin C, Cyclin D1, and Cyclin E1, was decreased. In the rescue experiments, levels of these proteins in cancer cells were restored due to the restoration of PSAT1. These findings suggested that microRNA-145-5p affected cell cycle via targeting PSAT1, and cell cycle pathway is reported to be closely associated with the proliferation of cancer cells.

Overall, this study highlighted that microRNA-145-5p inhibited PSAT1 level and cell proliferation in colon cancer. This newly discovered microRNA-145-5p/PSAT1 regulatory axis may offer new strategies for colon cancer management. In future studies, microRNA-145-5p may be employed to provide new breakthroughs in cancer diagnosis and treatment. Although the experimental design of this study is reasonable and the arguments are substantial, there are also some limitations. First, clinical tumor samples are required to analyze the correlation of microRNA-145-5p with clinical parameters to confirm its role in colon cancer metastasis. Second, the exact role of microRNA-145-5p in colon cancer proliferation, metastasis and downstream signaling pathways in vivo has not been elucidated, therefore, further in-depth research is needed to provide a theoretical basis for clinical practice.

## 5. Conclusion

In summary, our study disclosed that microRNA-145-5p was down-regulated in colon cancer, and microRNA-145-5p repressed proliferation and migration of colon cancer cells. Notably, our study revealed for the first time that microRNA-145-5p modulated colon cancer malignant progression in vitro via targeting PSAT1. These findings may provide new avenue for colon cancer treatment.

## Supplementary Material

Supplemental Material

## Data Availability

The data used to support the findings of this study are included within the article. The data and materials in the current study are available from the corresponding author on reasonable request.
